# Multiresolution Mutual Assistance Network for Cardiac Magnetic Resonance Images Segmentation

**DOI:** 10.1155/2022/5311825

**Published:** 2022-10-31

**Authors:** Shaolong Chen, Changzhen Qiu, Weiping Yang, Zhiyong Zhang

**Affiliations:** School of Electronics and Communication Engineering, Sun Yat-sen University, Shenzhen 518107, China

## Abstract

The automatic segmentation of cardiac magnetic resonance (MR) images is the basis for the diagnosis of cardiac-related diseases. However, the segmentation of cardiac MR images is a challenging task due to the inhomogeneity of MR images intensity distribution and the unclear boundaries between adjacent tissues. In this paper, we propose a novel multiresolution mutual assistance network (MMA-Net) for cardiac MR images segmentation. It is mainly composed of multibranch input module, multiresolution mutual assistance module, and multilabel deep supervision. First, the multibranch input module helps the network to extract local and global features more pertinently. Then, the multiresolution mutual assistance module implements multiresolution feature interaction and progressively improves semantic features to more completely express the information of the tissue. Finally, the multilabel deep supervision is proposed to generate the final segmentation map. We compare with state-of-the-art medical image segmentation methods on the medical image computing and computer-assisted intervention (MICCAI) automated cardiac diagnosis challenge datasets and the MICCAI atrial segmentation challenge datasets. The mean dice scores of our method in the left atrium, right ventricle, myocardium, and left ventricle are 0.919, 0.920, 0.881, and 0.960, respectively. The analysis of evaluation indicators and segmentation results shows that our method achieves the best performance in cardiac magnetic resonance images segmentation.

## 1. Introduction

Cardiovascular disease is one of the world's leading causes of death, and it kills more people each year from cardiovascular disease than from any other disease [1, 2]. In recent years, the number of patients with cardiovascular disease has increased sharply. The prevention and treatment of cardiovascular disease should attract public attention. With the development of modern medicine, in order to reduce the mortality rate and misdiagnosis rate of cardiovascular diseases, medical imaging technologies such as magnetic resonance imaging (MRI), computerized tomography (CT), and ultrasound (US) are widely used in the diagnosis and treatment of cardiovascular diseases. Cardiac MRI is currently recognized as the gold standard for evaluating the cardiac function, and MRI has the advantages of less harm to the human body and clear imaging [3–6]. The automatic segmentation of cardiac magnetic resonance (MR) images is the basis for the diagnosis of cardiac-related diseases. In general, the anatomy of the cardiac MR image includes the left ventricle, right ventricle, epicardium, endocardium, and myocardium. At present, the main segmentation method in clinical use is manual segmentation by doctors, which can obtain accurate results but is very time-consuming. The limitations of manual segmentation have motivated researchers to continue developing automatic segmentation methods for cardiac segmentation [7].

The current cardiac MR images segmentation methods can be mainly divided into traditional methods [8–10] and deep learning-based methods [11–15]. Traditional methods mainly include graph searching based on intensity [8], region growing [9], and active appearance models [10]. However, most of these traditional methods have problems such as complex design, poor versatility, and low segmentation accuracy. In recent years, deep learning has achieved great success in medical image processing [16–19]. Some researchers introduced deep learning into medical image segmentation. The deep learning-based method gradually replaces the traditional medical image segmentation method due to its good versatility, high segmentation accuracy, and high efficiency [20–23]. The proposal of UNet [24] is a milestone in medical image segmentation. Based on the U-shaped structure and skip connections, UNet fuses low-resolution information and high-resolution information and has been widely used for cardiac MR images segmentation. Li et al. [25] proposed a new multiscale feature attentive UNet for cardiac MR images segmentation and achieved excellent performance. Sharan et al. [26] combined feature pyramid network and UNet architecture to study the automatic segmentation of left ventricle, myocardium, and right ventricle. Sharan et al. [27] proposed a stack attention-based convolutional neural network approach for fully automatic segmentation from short-axis cardiac MR images. Cui et al. [28] added the direction field module, channel self-attention module, and selective kernel module to the UNet framework to improve the segmentation performance, and the segmentation experiments on cardiac MR images demonstrated the effectiveness of the improvements. Wang et al. [29] proposed an auto-weighted supervision framework to solve the problem of scar and edema segmentation in multisequence cardiac MR images although the existing cardiac MR images segmentation methods have achieved good results. However, the segmentation of cardiac MR images is still a challenging task due to the inhomogeneity of MR images intensity distribution and the unclear boundaries between adjacent tissues.

Recently, Fu et al. [30] proposed that a multiscale input layer constructs an image pyramid to achieve multiple level receptive field sizes for optic disc and optic cup segmentation. It is proved that multiscale input can improve the segmentation performance. Shi et al. [31] proposed a multiinput fusion network model based on multiscale input and feature fusion, which automatically extracts and fuses the features of different input scales to realize the detection of cardiac MR images. Chen et al. [32] proposed a T-based multiresolution input network, which achieved good performance in the field of medical image segmentation. Currently, the application of multiresolution input in medical image segmentation is less studied. There is still a lot of room for improvement in the existing methods. Firstly, the existing multiresolution input network only considers the fusion of multiresolution features at the encoder side but does not consider the fusion of multiresolution features at the decoder side. Second, the shallow features extracted from high-resolution images contain a lot of irrelevant background information, and existing methods do not consider how to suppress this irrelevant background information by utilizing deep features extracted from low-resolution images.

In this paper, we propose a novel multiresolution mutual assistance network (MMA-Net) for cardiac MR images segmentation. It is mainly composed of multibranch input module, multiresolution mutual assistance module, and multilabel deep supervision. First, the multibranch input module is responsible for feature extraction of input images with different resolutions. Each resolution input image has a separate feature extraction branch. The high-resolution input image branch is responsible for learning the local information of the image without worrying about the loss of global information because the extraction of global information is completed by the low-resolution input image branch. Similarly, the low-resolution input image branch is responsible for learning the global information of the image without worrying about the loss of local information. Second, the multiresolution mutual assistance module implements multiresolution feature interaction and progressively improves semantic features to more completely express the information of the tissue. Finally, the multilabel deep supervision is proposed to generate the final segmentation map. In addition, we designed the attention gate that utilizes global features extracted from low-resolution input images to suppress irrelevant background information from local features extracted from high-resolution input images. We compared with state-of-the-art medical image segmentation methods on the medical image computing and computer-assisted intervention (MICCAI) automated cardiac diagnosis challenge datasets (ACDC) [33] and the MICCAI atrial segmentation challenge datasets (ASC) [34]. The mean dice score of our method in the left atrium, right ventricle, myocardium, and left ventricle are 0.919, 0.920, 0.881, and 0.960, respectively. The analysis of evaluation indicators and segmentation results shows that our method achieves the best performance in cardiac magnetic resonance images segmentation.

The main contribution of this work can be summarized as follows:

1. A novel multiresolution mutual assistance network (MMA-Net) for cardiac MR images segmentation is proposed. It implements multiresolution feature interaction and progressively improves semantic features to more completely express the information of the tissue.
2. We designed the attention gate that utilizes global features extracted from low-resolution input images to suppress irrelevant background information from local features extracted from high-resolution input images.
3. A multilabel deep supervision is proposed, which can well handle the problem of inconsistent prediction results and labels caused by up sampling of small-scale feature layers in deep supervision.
4. Our method outperforms the existing six excellent medical image segmentation methods.

## 2. Method

The proposed multiresolution mutual assistance network (MMA-Net) is shown in Figure 1. It is mainly composed of multibranch input module, multiresolution mutual assistance module, and multilabel deep supervision. As shown in Figure 1, first, 2D medical images with resolutions of 224 × 224 and 112 × 112 are input to the multibranch input module to extract features, respectively. Second, these extracted features are then input to the multiresolution mutual assistance module for information interaction and progressively improves semantic features to more completely express the information of the tissue. Finally, the multilabel deep supervision to guide the learning of the network and the prediction result of *M*_*D*,1_ are used as the final result.

### 2.1. Multibranch Input Module

The multiresolution input has been shown to be effective in improving segmentation quality [30]. The current multiresolution input mostly adopts the structure of the shared encoder. The disadvantage of this structure is that it is difficult to balance the learning of local features and global features. If the receptive field of the convolution kernel in the convolutional layer is increased, the learning of global features can be enhanced, but some local features will be lost at the same time, and vice versa. Therefore, we adopted a multibranch structure with a separate encoder for each resolution input. The high-resolution input branch can learn the local information of the image without worrying about the loss of global information because the extraction of global information is done by the low-resolution input branch. Similarly, the low-resolution input branch is responsible for learning the global information of the image without worrying about the loss of local information. For the selection of the number of branches, after our experiments, we chose the dual-branch structure, as shown in Figure 1. For branch 1, its input is an image with a resolution of 224 × 224, and the output is the feature *M*_*E*,*i*_ (*i* = 1, 2, 3, 4, 5) of each encoding stage. For branch 2, its input is an image with a resolution of 112 × 112, and the output is the feature *N*_*E*,*j*_ (*j* = 2, 3, 4, 5, 6) of each encoding stage.

### 2.2. Multiresolution Mutual Assistance Module

After obtaining the features at each stage of the input image at different resolutions, our goal is to use this information to obtain better decoded features for final segmentation prediction. The input to multiresolution mutual assistance module is the features of each stage of the branch 1 and branch 2 encoders, including *M*_*E*,*i*_ (*i* = 1, 2, 3, 4, 5) and *N*_*E*,*j*_ (*j* = 2, 3, 4, 5, 6). The outputs are the features of each stage of the branch 1 and branch 2 decoders, including *M*_*D*,*i*_ (*i* = 1, 2, 3, 4) and *N*_*D*,*j*_ (*j* = 2, 3, 4). For each branch, the input to each decoder stage consists of the complementary features generated by the previous stage and the features of the corresponding encoder stage. The output of each stage of the decoder is calculated by the following formulas.

For branch 1,

(1) $$\begin{array}{c} \left\{\begin{array}{l} M_{D,i}=A\left(Up\left(F\left(M_{D,i+1},N_{D,i+1}\right)\right),M_{E,i}\right),i=1,2,3,\\ M_{D,4}=A\left(Up\left(F\left(Up\left(N_{E,6}\right),AG\left(Up\left(N_{E,6}\right),M_{E,5}\right)\right)\right),M_{E,4}\right). \end{array}\right. \end{array}$$

For branch 2,

(2) $$\begin{array}{c} \left\{\begin{array}{l} N_{D,j}=A\left(Up\left(F\left(M_{D,j+1},N_{D,j+1}\right)\right),N_{E,j}\right),j=2,3\text{,}\\ N_{D,4}=A\left(Up\left(F\left(Up\left(N_{E,6}\right),AG\left(Up\left(N_{E,6}\right),M_{E,5}\right)\right)\right),N_{E,4}\right)\text{.} \end{array}\right. \end{array}$$

Here, **Up** is the up sampling; **AG** is the attention gate; **A** is the attention feature selection; and **F** is the feature fusion.

#### 2.2.1. Attention Gate

In our network, branch 1 is mainly used to extract shallow local features, and branch 2 is mainly used to extract deep global features. Local features contain a large amount of detailed information of the target tissue, but they also introduce a lot of irrelevant background information. Global features contain information such as the location of the target tissue, and there is less detailed information, but there is also little irrelevant background information. Inspired by reference [35], we designed an attention gate that utilizes global features of the last stage (*N*_*E*,6_) of branch 2 to suppress the irrelevant background information of the local features of the last stage (*M*_*E*,5_) of branch 1. The structure of attention gate is shown in Figure 2.

#### 2.2.2. Attention Feature Selection

For each branch, the input to each decoder stage consists of the complementary features generated by the previous stage and the features of the corresponding encoder stage. The feature input from the encoder stage has shallower features than the corresponding complementary features. Therefore, we also designed to use complementary features to suppress the irrelevant background information of the corresponding encoder stage input features, and the attention feature selection is shown in Figure 3.

#### 2.2.3. Feature Fusion

It first concatenates multiple input features along the channel axis and then applies two 3 × 3 convolutional layers to the fusion result with the same number of output channels as a single input.

### 2.3. Multilabel Deep Supervision

In deep supervision, there are only labels of the same size as the original image. The prediction result of the last layer is the same as the scale of the label, and the loss can be calculated directly with the label. The prediction results of other small-scale feature layers are usually up sampling to the original image size, and then the loss is calculated with the labels. However, during the up sampling process, the prediction results become coarse, which may lead to inconsistencies between the prediction results and the labels. To solve this problem, we propose a multilabel deep supervision.  Figure 4 shows the deep supervision and multilabel deep supervision of *M*_*D*,1_ and *M*_*D*,4_ layers. As shown in Figure 4(a), in the deep supervision, the consistency between *M*_*D*,1_ results and labels is good, but the consistency between up sampling and labels is poor in *M*_*D*,4_ results, which may cause the network to learn wrong information. As shown in Figure 4(b), in the multilabel deep supervision, each scale feature layer has a label that is consistent with its feature map size. The results are consistent with the label, which can well guide the network learning.

We have seven output prediction maps and the total loss function is a simple addition of the loss functions of these seven output prediction maps. For each output prediction map, we considered the combination of binary cross-entropy and dice loss as

(3) $$\begin{array}{c} L=L_{BCE}+L_{DICE}\text{.} \end{array}$$

Here,

(4) $$\begin{array}{c} L_{BCE}=\underset{x,y}{\sum }G_{x,y}*\;\log\left(Q_{x,y}\right)+\left({1-G}_{x,y}\right)*\;\log\;\left(1-Q_{x,y}\right)\text{,}\\ L_{DICE}=1-\frac{2\underset{x,y}{\sum }G_{x,y}{*Q}_{x,y}}{\underset{x,y}{\sum }\left(G_{x,y}+Q_{x,y}\right)}\text{,} \end{array}$$

where *L*_BCE_ and *L*_DICE_ represent the binary cross-entropy loss and dice loss, respectively. *G*_*x*,*y*_ ∈ {0,1} is the area label at position (x, y), and *Q*_*x*,*y*_ ∈ [0,1] is the area value at position (x, y) in output prediction.

## 3. Experiments

### 3.1. Datasets, Preprocessing, Implementation Details, and Evaluation Metrics

#### 3.1.1. Datasets and Preprocessing

We evaluated our method at the medical image computing and computer-assisted intervention (MICCAI) automated cardiac diagnosis challenge (ACDC) [33] and the MICCAI atrial segmentation challenge (ASC) [34]. The ACDC has cardiac MR images for 150 cases, but only 100 cases are annotated (right ventricle, myocardium, and left ventricle), and we only use the 100 annotated cases. The ASC has 154 cardiac MR images, all annotated. For all datasets, we additionally cropped input images at their centers to make their size 224 × 224 pixels. In addition, we performed max-min normalization (0–1) for each case. For both the ACDC and ASC datasets, we augmented the training set by slightly translating, scaling, and rotating. We evaluated the performance of each model by 5-fold cross-validation.

#### 3.1.2. Implementation Details

Each model runs on four RTX 3090 cards. We trained our network in the multilabel deep supervision way. All models are trained with the Adam optimizer with batch size 32, learning rate 5∗10^−4^, momentum 0.9, weight decay 1∗10^−4^, and max-epoch 1000. The early stopping is set to 20. For each branch, we use VGG19 as the backbone network to extract features.

#### 3.1.3. Evaluation Metrics

We measured the accuracy of segmentation by the dice similarity coefficient (dice), specificity , sensitivity, and F1-score (F1) by

(5) $$\begin{array}{c} di\;ce=\frac{2*\left(A\cap B\right)}{A\cup B}\text{,}\\ \begin{array}{c} specificity=\frac{TN}{TN+FP},\\ sensitivity=\frac{TP}{TP+FN},\\ F1=\frac{2*TP}{2*TP+FP+FN}, \end{array} \end{array}$$

where A and B represent prediction result and ground truth, respectively. TP, TN, FP, and FN represent the number of true positives, true negatives, false positives, and false negatives, respectively.

### 3.2. Ablation Experiments and Analyses

#### 3.2.1. Number of Branches

We analyzed the influence of the number of branches in the network on the segmentation accuracy in the ACDC and ASC, which includes (a) *Num* = 1 (the input image size is 224 × 224), (b) *Num* = 2 (the input image sizes are 224 × 224 and 112 × 112, respectively), (c) *Num* = 3 (the input image sizes are 224 × 224, 112 × 112 and 56 × 56, respectively), and (d) *Num* = 4 (the input image sizes are 224 × 224, 112 × 112, 56 × 56 and 28 × 28, respectively). The results are shown in Tables 1 and 2. According to our network structure rules, when *Num* = 5, branch 5 will have no decoder stage; therefore, we do not compare the case of *Num* ≥ 5. As shown in Tables 1 and 2, when *Num* = 2, the segmentation performance of the network is the best, so we finally chose the dual-branch network structure.

#### 3.2.2. Multiresolution Mutual Assistance Module

We analyzed the influence of the multiresolution mutual assistance module in the network on the segmentation accuracy in the ACDC and ASC, which includes (a) unidirectional fusion mode (UFM), (b) two-way fusion mode (TFM), and (c) multiresolution mutual assistance module (MMAM). The results are shown in Tables 3 and 4. As shown in Tables 3 and 4, compared with other modes, our multiresolution mutual assistance module achieves better performance.

#### 3.2.3. Multilabel Deep Supervision

We analyzed the influence of the multilabel deep supervision in the network on the segmentation accuracy in the ACDC and ASC, which includes (a) deep supervision (DS) and (b) multilabel deep supervision (MLDS). The results are shown in Tables 5 and 6. As shown in Tables 5 and 6, compared with deep supervision, our multilabel deep supervision achieves better performance. This is because in deep supervision, the results of small-scale feature layers are inconsistent with the labels, causing the network to learn wrong information. Our multilabel deep supervision has labels of corresponding sizes for each scale feature layer. The results are consistent with the label, which can well guide the network learning.

### 3.3. Comparison with State-of-the-Art Methods and Discussion

In this section, we compared the proposed MMA-Net with previous state-of-the-art medical image segmentation methods on the ACDC [33] and the ASC [34].

#### 3.3.1. Quantitative Comparison

Tables 7 and 8 show the segmentation results on the ACDC and the ASC, respectively. As shown in Tables 7 and 8, our method achieves the best performance for most of the metrics on the ACDC and the ASC. Especially in the dice, as a key indicator for evaluating the performance of medical image segmentation, our method has a great improvement compared with other methods. The specificity of all methods is close to 1.000 because the background is the majority, and most of the background is easily classified. Our method may be more sensitive to tissue, misclassifying many backgrounds as tissue, which may be the reason why our method does not achieve optimal performance in terms of specificity. Sensitivity is another important metric to evaluate the performance of medical image segmentation, and our method achieves a large performance improvement on RV, Myo, and LV, and a certain performance improvement on LA as well. F1 is a relatively comprehensive evaluation index for medical image segmentation performance, and our method has a certain degree of improvement compared with other methods.  Figure 5 shows the change in loss and dice of our method on the ACDC (RV tissue). As the number of iterations increases, the loss function converges rapidly, proving that our network structure and training parameter design are reasonable.

#### 3.3.2. Qualitative Comparison

Figure 6 shows the visualizations on the right ventricle (RV), myocardium (Myo), left ventricle (LV), and left atrium (LA). As shown in Figure 6, compared with other methods, our method shows significant improvement in segmentation performance. For the RV tissue, our method can localize the tissue well and segment the edges of the tissue well. For the Myo tissue, only our method formed complete rings, and none of the other methods formed complete rings. LV is an easy tissue to segment, but other methods still have some segmentation failures. Our method can segment the LV tissue more perfectly. LA is a difficult tissue to segment, and other methods are generally effective in segmenting the details of LA tissue. Our method can better segment the details of LA.

## 4. Conclusion

In this paper, a novel multiresolution mutual assistance network (MMA-Net) for cardiac MR images segmentation is proposed. It implements multiresolution feature interaction and progressively improves semantic features to more completely express the information of the tissue. We compare with state-of-the-art medical image segmentation methods on the ACDC and the ASC. The mean dice score of our method in the left atrium, right ventricle, myocardium, and left ventricle are 0.919, 0.920, 0.881, and 0.960, respectively. The analysis of evaluation indicators and segmentation results shows that our method achieves the best performance in cardiac magnetic resonance images segmentation.

## Figures and Tables

**Figure 1:** The proposed multiresolution mutual assistance network (MMA-Net).

**Figure 2:** Attention gate.

**Figure 3:** Attention feature selection.

**Figure 4:** The deep supervision and multilabel deep supervision of the *M*_*D*,1_ and *M*_*D*,4_ layers. (a) Deep supervision. (b) Multilabel deep supervision.

**Figure 5:** The change in loss and dice of our method on the ACDC (RV tissue).

**Figure 6:** Qualitative comparisons with state-of-the-art methods.

**Table 1:** The influence of the number of branches in the network on the segmentation accuracy in the ACDC.

	*Num* = 1	*Num* = 2	*Num* = 3	*Num* = 4
Dice	0.897	**0.920**	0.911	0.908
Specificity	0.999	**0.999**	0.999	0.999
Sensitivity	0.891	**0.915**	0.902	0.900
F1	0.899	**0.920**	0.911	0.908

The best performance is shown in bold.

**Table 2:** The influence of the number of branches in the network on the segmentation accuracy in the ASC.

	*Num* = 1	*Num* = 2	*Num* = 3	*Num* = 4
Dice	0.909	**0.919**	0.914	0.912
Specificity	0.995	**0.996**	0.996	0.995
Sensitivity	0.911	**0.917**	0.914	0.913
F1	0.911	**0.920**	0.915	0.913

The best performance is shown in bold.

**Table 3:** The influence of the multiresolution mutual assistance module in the network on the segmentation accuracy in the ACDC.

	UFM	TFM	MMAM
Dice	0.908	0.909	**0.920**
Specificity	0.999	0.999	**0.999**
Sensitivity	0.900	0.899	**0.915**
F1	0.908	0.911	**0.920**

The best performance is shown in bold.

**Table 4:** The influence of the multiresolution mutual assistance module in the network on the segmentation accuracy in the ASC.

	UFM	TFM	MMAM
Dice	0.911	0.910	**0.919**
Specificity	0.995	0.995	**0.996**
Sensitivity	0.913	0.912	**0.917**
F1	0.911	0.910	**0.920**

The best performance is shown in bold.

**Table 5:** The influence of the multilabel deep supervision in the network on the segmentation accuracy in the ACDC.

	DS	MLDS
Dice	0.915	**0.920**
Specificity	0.999	**0.999**
Sensitivity	0.908	**0.915**
F1	0.915	**0.920**

The best performance is shown in bold.

**Table 6:** The influence of the multilabel deep supervision in the network on the segmentation accuracy in the ASC.

	DS	MLDS
Dice	0.916	**0.919**
Specificity	0.996	**0.996**
Sensitivity	0.915	**0.917**
F1	0.917	**0.920**

The best performance is shown in bold.

**Table 7:** Comparison with state-of-the-art methods on the ACDC.

		UNet [24]	Att-UNet [35]	UNet++ [36]	UNet3+ [37]	TransUNet [38]	Swin-UNet [39]	Ours
Dice	RV	0.892	0.895	0.900	0.905	0.901	0.841	**0.920**
	Myo	0.861	0.851	0.858	0.854	0.845	0.775	**0.881**
	LV	0.939	0.940	0.936	0.947	0.942	0.909	**0.960**

Specificity	RV	0.998	0.999	0.999	0.999	0.999	0.997	**0.999**
	Myo	0.999	0.998	**0.999**	0.999	0.998	0.997	0.998
	LV	0.999	0.999	0.999	0.999	0.999	0.999	**0.999**

Sensitivity	RV	0.891	0.885	0.894	0.900	0.899	0.855	**0.909**
	Myo	0.852	0.849	0.840	0.843	0.868	0.800	**0.883**
	LV	0.929	0.928	0.931	0.939	0.950	0.894	**0.953**

F1	RV	0.894	0.898	0.902	0.907	0.903	0.845	**0.921**
	Myo	0.863	0.854	0.859	0.856	0.847	0.777	**0.881**
	LV	0.941	0.942	0.939	0.949	0.945	0.910	**0.960**

The best performance is shown in bold.

**Table 8:** Comparison with state-of-the-art methods on the ASC.

		UNet [24]	Att-UNet [35]	UNet++ [36]	UNet3+ [37]	TransUNet [38]	Swin-UNet [39]	Ours
Dice	LA	0.909	0.908	0.907	0.907	0.904	0.876	**0.919**
Specificity	LA	0.995	0.995	0.996	0.995	0.995	0.994	**0.996**
Sensitivity	LA	0.911	0.914	0.905	0.911	0.902	0.887	**0.917**
F1	LA	0.911	0.911	0.911	0.911	0.908	0.886	**0.920**

The best performance is shown in bold.

## Data Availability

The data used to support the findings of this study are available from the corresponding author upon request.
